The article "TGFβ3 recruits endogenous mesenchymal stem cells to initiate bone regeneration" was retracted in 2022. Reasons: duplicated images; original data or images not available; unreliable results or conclusions.

# TGFβ3 recruits endogenous mesenchymal stem cells to initiate bone regeneration

**DOI:** 10.1186/s13287-017-0693-0

**Published:** 2017-11-10

**Authors:** Moyuan Deng, Tieniu Mei, Tianyong Hou, Keyu Luo, Fei Luo, Aijun Yang, Bo Yu, Hao Pang, Shiwu Dong, Jianzhong Xu

**Affiliations:** 1 National & Regional United Engineering Lab of Tissue Engineering, Department of Orthopaedics, Southwest Hospital, the Third Military Medical University, Chongqing, China; 2 Department of Biomedical Materials Science, College of Biomedical Engineering, Third Military Medical University, Chongqing, China; 3 Department of Surgery, Fuzhou Mawei Naval Hospital, Fujian, China

**Keywords:** TGFβ3, Recruitment, Mesenchymal stem cell, Vascular cells, MCP1

## Abstract

**Background:**

The recruitment of a sufficient number of endogenous mesenchymal stem cells (MSCs) is the first stage of in-situ tissue regeneration. Transforming growth factor beta-3 (TGFβ3) could recruit stem or progenitor cells and endothelial cells to participate in tissue regeneration. However, the mechanism of TGFβ3 recruiting MSCs toward bone regeneration has remained obscure.

**Methods:**

We estimated the promigratory property of TGFβ3 on human bone marrow MSCs (hBMSCs) cocultured with the vascular cells (human umbilical artery smooth muscle cells or human umbilical vein endothelial cells) or not by Transwell assay. After the addition of the inhibitor (SB431542) or Smad3 siRNA, the levels of MCP1 and SDF1 in coculture medium were tested by ELISA kit, and then the migratory signaling pathway of hBMSCs induced by TGFβ3 was investigated by western blot analysis. In vivo, a 2-mm FVB/N mouse femur defect model was used to evaluate chemokine secretion, endogenous cell homing, and bone regeneration induced by scaffolds loading 1 μg TGFβ3 through qPCR, immunofluorescent staining, immunohistochemical analysis, and Micro-CT, compared to the vehicle group.

**Results:**

TGFβ3 (25 ng/ml) directly showed a nearly 40% increase in migrated hBMSCs via the TGFβ signaling pathway, compared to the vehicle treatment. Then, in the coculture system of hBMSCs and vascular cells, TGFβ3 further upregulated nearly 3-fold MCP1 secretion from vascular cells in a Smad3-dependent manner, to indirectly enhance nearly more than 50% of migrated hBMSCs. In vivo, TGFβ3 delivery improved MCP1 expression by nearly 7.9-fold, recruited approximately 2.0-fold CD31^+^ vascular cells and 2.0-fold Sca-1^+^ PDGFR-α^+^ MSCs, and achieved 2.5-fold bone volume fraction (BV/TV) and 2.0-fold bone mineral density, relative to TGFβ3-free delivery.

**Conclusions:**

TGFβ3, as a MSC homing molecule, recruited MSCs to initiate bone formation in the direct-dependent and indirect-dependent mechanisms. This may shed light on the improvement of MSC homing in bone regeneration.

The article "TGFβ3 recruits endogenous mesenchymal stem cells to initiate bone regeneration" was retracted in 2022. Reasons: duplicated images; original data or images not available; unreliable results or conclusions.

## Background

Traumatic bone injury, tumor resection, and osteitis cause a large bone defect, and improving in-situ bone regeneration is vital to heal bone defects. From the perspective of in-situ tissue regeneration, utilizing the body’s endogenous healing capacity requires the recruitment of mesenchymal stem cells (MSCs) to an injury site [1–4]. The mode of recruitment is directional migration in response to a gradient of soluble chemoattractants, including chemokines and proinflammatory cytokines [5]. Stromal cell-derived factor-1 (SDF-1) has been widely discussed as a potent chemoattractant, which can recruit endogenous MSCs to increase the bone volume fraction (BV/TV) and produce a significantly higher bone mineral density (BMD) via the SDF-1/CXC chemokine receptor 4 (CXCR4) axis [4, 6]. What is more, monocyte chemoattractant protein 1 (MCP1) and its CCL2–CCR2 axis play an important role in endogenous MSC homing during the early phase of fracture healing [7]. Last of all, transforming growth factor beta-1 (TGFβ1) also has an excellent effect on improving MSC homing [8, 9].

The TGFβ superfamily plays major roles in development, homeostasis, and regeneration of bone tissue [10]. Some studies have shown that injury-activated TGFβ members control the migration of MSCs [9, 11, 12]. Although the promigratory property of TGFβ1 and TGFβ2 on MSCs has been reported, the role and mechanism of TGFβ3 on the recruitment of MSCs toward bone formation are unknown [9, 13].

MSCs are recruited to the injury site by homing mainly through the vascular network [14]. TGFβ3 could recruit vascular cells and promote the function of endothelial cells and neovascularization [15]. Additionally, endothelial cells have been demonstrated to express some chemokines, such as MCP1, which is reported to be essential for recruitment of human bone marrow-derived MSCs (hBMSCs) [7, 16–18]. If TGFβ3 has a positive effect on chemokine expression from vascular cells, it is logical to assume that TGFβ3 would improve MSC recruitment. The fate of homing MSCs is mediated by environmental cues, including from the TGFβ, BMP, and Wnt signaling pathways. These environmental cues, in the early stage of fracture, could upregulate TEAD2/GTF2I motifs levels, or downregulate JARID1B histone demethylase, which results in an increase of RUNX2 expression, a key transcription factor for MSC osteogenesis [19, 20]. Thus, the MSCs, which are recruited toward the bone injury site and impacted by these environmental cues, have been reported to promote bone formation [21, 22].

In this study, we estimated the direct promigratory potency and mechanism of TGFβ3 in hBMSCs. Furthermore, the effect of vascular cells on TGFβ3-induced migration of hBMSCs was estimated. Thirdly, we discussed the signaling pathway of TGFβ3-induced migration of hBMSCs cocultured with vascular cells or not. Finally, the role of TGFβ3 delivery in recruiting endogenous MSCs toward bone formation was evaluated in a 2-mm FVB/N mouse femur defect model.

The article "TGFβ3 recruits endogenous mesenchymal stem cells to initiate bone regeneration" was retracted in 2022. Reasons: duplicated images; original data or images not available; unreliable results or conclusions.

## Methods

### Isolation and culture of bone marrow-derived MSCs

The protocols to isolate hBMSCs were approved by the Institutional Ethics Committee at the Southwest Hospital of the Third Military Medical University. The volunteers who donated bone marrow signed informed consent forms. The protocols to isolate and characterize hBMSCs were described in our previous study [23]. The hBMSCs were isolated by density gradient centrifugation. hBMSCs were cultured in DMEM/F12 (HyClone Laboratories, UT, USA) with 10% fetal bovine serum (FBS; Gibco, USA), 100 U/ml penicillin, and 0.1 mg/ml streptomycin. The cells from passages 3-5 were used for the experiments described in this study.

### Culture of vascular smooth muscle cells and vascular endothelial cells

Human umbilical artery smooth muscle cells (hUASMCs) and human umbilical vein endothelial cells (hUVECs) were from ScienCell (CA, USA). hUASMCs were cultured in smooth muscle cell medium (ScienCell Inc., CA, USA), and hUVECs were cultured in endothelial cell medium (ScienCell Inc., CA, USA).

### Small interfering RNA transfection

Predesigned double-stranded small interfering RNAs (siRNAs) from Integrated DNA Technologies were used; 30 pmol of human Smad3 silencing RNA (siRNA) (Santa Cruz Biotechnology, TX, USA) or nonspecific control siRNA (Santa Cruz Biotechnology) were transfected into hBMSCs using Lipofectamine RNAi (Thermo Fisher Scientific) according to the manufacturer’s protocol. Then, after 48 hours of transfection, cells were treated with TGFβ3 or vehicle control. FITC-conjugated control siRNA (Santa Cruz) was used to test for transfection efficiency, and approximately 80-90% of cells were transfected with siRNA.

### Cell migration

#### Single cell culture system

Approximately 5 × 10^4^ hBMSCs were seeded with DMEM/F12 medium on the upper Boyden chambers of 24-well plates (8 μm; Corning, Inc., USA) and the culture medium with different concentrations of TGFβ3 and 2% FBS was placed into the lower chambers. After incubating plates for 6 hours at 37 °C, the cells of the upper chamber were fixed, stained with 0.5% crystal violet dye, and removed with a cotton swab. The cells migrating to the lower surface were photographed and counted under a microscope. For TβRI/II signaling pathway inhibition, hBMSCs were pretreated with SB431542 (15 μM; Selleckchem Inc., TX, USA) for 1 hour prior to the growth factor administration.

The article "TGFβ3 recruits endogenous mesenchymal stem cells to initiate bone regeneration" was retracted in 2022. Reasons: duplicated images; original data or images not available; unreliable results or conclusions.

#### Coculture system of hBMSCs and vascular cells

Approximately 5 × 10^4^ hBMSCs were seeded with DMEM/F12 medium on the upper Boyden chambers of 24-well plates (8 μm; Corning, Inc.) and approximately 5 × 10^4^ vascular cells (hUASMCs or hUVECs) were seeded with the culture medium with the different concentrations of TGFβ3 and 2% FBS on the lower chambers. After incubating plates for 6 hours at 37 °C, hBMSC migration was assessed using the crystal violet dye method.

### TGFβ3 delivery

In vitro, TGFβ3 (Pepro Tech Inc., NJ, USA) was prepared at different concentrations (5-100 ng/ml) of culture medium to assess cell migration and protein levels. On the other hand, in vivo, 100 μl TGFβ3 at a dose of 10 μg/ml was adsorbed in absorbable gelatin sponges (Jinling Pharmaceutical Company, Jiangsu, China) to prepare the scaffold loading TGFβ3.TGFβ3-free scaffold was used as a vehicle control [9].

### Western blotting analysis

To estimate the signaling pathway of vascular cells (hUASMCs or hUVECs) stimulated with TGFβ3 in the coculture system of hBMSCs and vascular cells, approximately 2 × 10^5^ hBMSCs were seeded on the upper Boyden chambers of six-well plates (0.4 μm; Corning, Inc.), and 2 × 10^5^ vascular cells (hUASMCs or hUVECs) were seeded on the lower chambers. The cells of the coculture system were incubated in culture medium containing 25 ng/ml TGFβ3 for 6 or 24 hours at 37 °C. Total protein was extracted with 100 μl RIPA lysis buffer (P0013B; Beyotime, Jiangsu, China), subjected to SDS-PAGE, transferred onto nitrocellulose membranes (Millipore, Billerica, USA), and probed with specific primary Abs against p-Smad3 (Cell Signaling Technology, USA), Smad3 (Santa Cruz Biotechnology), or GAPDH (Beyotime) at 1:500 dilution overnight at 4 °C. Immunoreactive protein bands were visualized using ECL chemiluminescence detection plus a western blot detection system (Bio-Rad, USA). The intensity ratio was the relative expression of p-Smad3, Smad3, TβRI, and TβRII normalized to GAPDH.

### ELISA

Vascular cells were treated by culture medium containing 25 ng/ml TGFβ3 or PBS for 24 hours. The culture medium was collected and the concentrations of MCP1 and SDF1 were measured with the BCA protein assay kit, and the cytokine concentration was measured with ELISA kits (ELH-Human SDF1 alpha, ELH-Human MCP1; RayBiotech, USA).

### Animal surgical procedure and experimental design

Eight-week-old FVB/N mice (weighing approximately 25–30 g, from the Animal Experiment Centre of Southwest Hospital of China) underwent a femoral osteotomy. The established surgical procedure has been reported previously [24]. Briefly, FVB/N mice were anesthetized and stabilized with fixation plates. The unilateral 2-mm segmental defects with removal of the periosteum were created in each mouse. The different scaffolds were transplanted into the bone defects. The wounds were closed using a standard surgical procedure. Mice were randomly assigned to two groups: the vehicle group (*n* = 24) and the TGFβ3 group (*n* = 24). To test the host MSCs, scaffold samples were retrieved and used for immunofluorescence colonization staining at 7 days postoperatively. To test vascularization of regenerated tissue, scaffold samples were retrieved and used for immunohistochemical analysis at 7 days postoperatively. At 8 weeks post operation, the development of new bone in the defects was monitored by micro-CT and the healing capacity of different treatments was further confirmed by the histology assessment.

The article "TGFβ3 recruits endogenous mesenchymal stem cells to initiate bone regeneration" was retracted in 2022. Reasons: duplicated images; original data or images not available; unreliable results or conclusions.

### Quantitative real-time PCR

Scaffolds were retrieved at 3, 7, and 14 days. The total RNA of treated cells was extracted with TRIzol reagent (TaKaRa, Shiga, Japan) and reverse transcribed with PrimeScript™-RT reagent kit (TaKaRa) according to the manufacturer’s instructions. Real-time PCR was performed using 2 × SYBR Green PCR Master Mix (Applied Biosystems, USA) on a Real-Time PCR System (Applied Biosystems 7500, USA). All of the primer sequences (Sangon Biotech Co., Ltd, Shanghai, China) were designed using primer 5.0 software. The following primer sets were used: *MCP1*, forward 5′-CTCGCCTCCAGCATGAAAGTCTC-3′ and reverse 5′-TGGGGTCAGCACAGATCTCCTTG-3′; and *β-ACTIN*, forward 5′-GCACAGAGCCTCGCCTTT-3′ and reverse 5′-CGCCCACATAGGAATCCTTC-3′. The relative expression of MCP1 was calculated using the 2^− *ΔΔ*Ct^ method, with β-actin as a reference gene.

### Immunofluorescent staining

The scaffolds retrieved at 7 days in vivo were embedded in optimal cutting temperature compound, and snap frozen at –20 °C. Sections (8-μm thick) were held overnight at 4 °C with primary antibodies against Sca-1 (1:500, 7 H4L3; Invitrogen, CA, USA) and PDGFR-α (1:500; Invitrogen) [25]. As appropriate, secondary antibodies labeled with Alexa Fluor 488 (1:100, donkey anti-rabbit) or Cy3 (1:100, goat anti-rat; ZSGB-BIO, Beijing, China) were used, and DAPI was used to stain nuclei. Fluorescence images were acquired using a Two Photon Laser Scanning System (LSM 510 NLO; Zeiss, Oberkochen, Germany). Endogenous cells and Sca-1^+^PDGFR-α^+^ MSCs migrating into the defect site were quantified at day 7 based on immunofluorescent images. A total of three images per animal distributed within the defect area, with 800× magnification, were analyzed.

The article "TGFβ3 recruits endogenous mesenchymal stem cells to initiate bone regeneration" was retracted in 2022. Reasons: duplicated images; original data or images not available; unreliable results or conclusions.

### Micro-CT

New bone formation on weeks 4 and 8 was evaluated with micro-CT (Skyscan, Antwerp, Belgium). The regenerated femora with removal of muscle in 4% paraformaldehyde were scanned with the following settings: voxel size 10.0 μm, voltage 65 kV, current A, and exposure time 280 ms. The data were subsequently analyzed and imaged using CT Analyser software (version 1.16.1.0, Skyscan 1272; Bruker Microct, Kontich, Belgium). 3D pictures were made with CTvox software (version 3.2.0r1294, Skyscan 1272; Bruker Microct) [26]. In the zone of the regenerated bone with the defects, the elliptical region of interest (ROI) was setted as 80 × 55 pixels, and the number of slices and predetermined threshold was from 264 to 1500 mg HA/cm^3^. The relative bone volume per tissue volume (BV/TV) and BMD of the regenerated bone within the defects were calculated using CTvox software (version 3.2.0r1294; Skyscan) [27].

### Immunohistochemical analysis

The femur samples were retrieved. The muscle and soft tissue were stripped off. The samples were then fixed in 4% buffered paraformaldehyde, decalcified in 10% EDTA, embedded in paraffin, and sectioned at 4–6 mm thickness. The slides were used for immunohistochemistry of CD31 (the endothelial marker). The slides of deparaffinized and rehydrated tissue sections were incubated in 3% H_2_O_2_ solution for 10 min to extinguish endogenous peroxidase activity and then washed with PBS. For antigen retrieval, the sections were irradiated in a microwave oven for 5 min in pH 6.0 citrate buffer. The primary antibody for CD31 (1:20 dilution; Santa Cruz) was applied overnight at 4 °C followed by incubation with biotinylated anti-mouse IgG for 30 min. The sections were counterstained with DAB for 3 min. Mayer′s hematoxylin was used for counterstaining [28].

### Statistical analysis

One-way ANOVA followed by Tukey’s test was utilized to determine the statistical significance of the differences in TGFβ3-induced hBMSC migration and western blot analysis. Two-way ANOVA followed by Sidak’s multiple comparisons test was performed to determine the statistical significance of the hBMSC migration in the coculture system, quantitative real-time PCR (qRT-PCR), and micro-CT data. Data are expressed as the means ± SD. The results are displayed as the mean ± standard deviation for *n* ≥ 3 samples per group in all cases, unless otherwise indicated. For both the ANOVA and post-hoc tests, differences were considered significant if *P* < 0.05.

## Results

### TGFβ3 improved hBMSC migration via the TGFβ signaling pathway

Many studies have demonstrated TGFβ1 could improve hBMSC migration [8, 10]. However, the role of TGFβ3 in hMSC migration has rarely been reported. Thus, we first evaluated whether recombinant TGFβ3 could directly stimulate hBMSC migration in vitro. The Transwell assay showed that TGFβ3 promoted hBMSC migration in a dose-dependent manner. At 25 ng/ml of TGFβ3, the number of migrated cells reached a peak and increased nearly 39.0 ± 9.5% more than that of the vehicle control (0 ng/ml) (*P* < 0.01; Fig. 1a).

The article "TGFβ3 recruits endogenous mesenchymal stem cells to initiate bone regeneration" was retracted in 2022. Reasons: duplicated images; original data or images not available; unreliable results or conclusions.

**Fig. 1:** Transwell assay for TGFβ3-induced hBMSC migration. **a** Analysis for migrated hBMSCs induced by 0 and 25 ng/ml TGFβ3 after 24-hour incubation. **b** Analysis for migrated hBMSCs induced by 0 and 25 ng/ml TGFβ3 with the pretreatment of inhibitor for TβRI/II. **c** Expression of TβRII in hBMSCs induced by TGFβ3 assessed by western blot analysis. Migrated cells were stained purple with crystal violet. Scale bar: 100 μm. *P < 0.05, **P < 0.01. TGFβ3 transforming growth factor beta-3, SB SB431542

As is well known, TGFβ could exert its cellular effects via TGFβ signals [15]. TGFβ signals act through serine/threonine kinase receptors known as TGFβ type II receptor (TβRII) and type I (TβRI). When the TGFβ ligand binds to TβRII, it recruits TβRI to form a heteromeric complex. TGFβ phosphorylates Tgfbr2/1, activating the receptor, which then activates downstream targets. Smad2 or Smad3 are phosphorylated by Tgfbr1. Phospho-Smad2 or 3 then associates with Smad4, leading to the transcription of downstream genes [10, 29–31]. In the present study, SB431542 completely inhibited the expression of TβRII and blocked TGFβ3-induced hBMSC migration, indicating that TGFβ3 promoted hBMSC migration through the TGFβ signaling pathway (*P* < 0.05 for TGFβ3 vs. Vehicle, *P* < 0.01 for TGFβ3 vs. TGFβ3+SB; Fig. 1b, c).

### The promigratory potential of TGFβ3 on hBMSCs was enhanced by vascular cells

MSCs are recruited to the injured sites by the vascular network [1]. Vascular cells play an important role in cell migration [9, 13, 15]. Thus, we investigated whether vascular cells would affect TGFβ3-induced hBMSC migration. The coculture system of MSCs and vascular cells was established (Fig. 2a). Vascular cells could strikingly increase the number of migrated hBMSCs. The number of migrated hBMSCs in the coculture system increased nearly 1.0 ± 0.3-fold and 1.5 ± 0.4-fold relative to the culture system without hUASMCs or hUVECs (*P* < 0.01 for the hUASMC system, *P* < 0.005 for the hUVEC system; Fig. 2a). In the coculture system of hBMSCs and hUVECs, a low concentration of 10 or 25 ng/ml of TGFβ3 greatly enhanced hBMSC chemotaxis, in which the number of migrated hBMSCs at 25 ng/ml in the TGFβ3 group increased 52.1 ± 13.6% relative to the vehicle group (*P* < 0.001 for 0 ng/ml vs 10 ng/ml, *P* < 0.005 for 0 ng/ml vs 25 ng/ml; Fig. 2b, d). On the other hand, in the coculture system of hBMSCs and hUASMCs, the number of migrated hBMSCs at 25 ng/ml in the TGFβ3 group increased 35.4 ± 10.1% (*P* < 0.05 for 0 ng/ml vs 25 ng/ml; Fig. 2c, d). Interestingly, the MSCs cocultured with hUVECs might have a stronger response to TGFβ3 stimulation than MSCs cocultured with hUASMCs (Fig. 2d).

The article "TGFβ3 recruits endogenous mesenchymal stem cells to initiate bone regeneration" was retracted in 2022. Reasons: duplicated images; original data or images not available; unreliable results or conclusions.

**Fig. 2:** Transwell assay for hBMSC migration. **a** Analysis for the migration of hBMSCs with or without hUVECs and hUASMCs. **b** In the coculture system of hBMSCs and hUASMCs, representative light photomicrographs of migrated hBMSC induced by 0-100 ng/ml TGFβ3 after 24-hour incubation. **c** In the coculture system of hBMSCs and hUVECs, representative light photomicrographs of migrated hBMSCs induced by 0-100 ng/ml TGFβ3 after 24-hour incubation. **d** Quantitative analysis of migrated cell density for (**c**) and (**d**). Migrated cells were stained purple with *crystal violet*. Scale bar: 100 μm. *P < 0.05, **P < 0.01, ***P < 0.005, ***P < 0.001. hUASMC human umbilical artery smooth muscle cell, hUVEC human umbilical vein endothelial cell, MSC mesenchymal stem cell, TGFβ3 transforming growth factor beta-3

### TGFβ3 upregulated MCP1 secretion from vascular cells

The addition of vascular cells remarkably upregulated the TGFβ3-induced hBMSC chemotaxis (Fig. 2a). The results might be due to the change of chemokine secretion in the coculture system. The ELISA results showed that TGFβ3 notably upregulated the secretion of MCP1 in the coculture system, but not SDF1, which has been reported to be involved in the recruitment of MSCs (Fig. 3a) [17, 28]. In 25 ng/ml TGFβ3, the expression of MCP1 in the hBMSC and hUASMC/hUVEC system increased 34.5.3 ± 3.7% and 78.4 ± 8.9%, respectively (*P* < 0.001 for hUVECs, *P* < 0.01 for hUASMCs; Fig. 3a). What is more, we investigated which cell was responsible for the increase of MCP1 secretion in the coculture system. The culture medium of hBMSCs, hUASMCs, and hUVECs was measured using an MCP1 ELISA kit. The results showed that TGFβ3 did not improve the secretion of MCP1 in the hBMSC group, but increased MCP1 secretions by 34.5 ± 3.7% and 78.4 ± 8.9% from hUASMCs and hUVECs (*P* < 0.001 for hUVECs, *P* < 0.01 for hUASMCs; Fig. 3b).

**Fig. 3:** TGFβ3 upregulated MCP1 secretion from vascular cells by TβRII/Smad3 signaling. **a** Secretion of MCP1 and SDF1 from vascular cells in the coculture system hBMSCs and vascular cells with TGFβ3. **b** Secretion of MCP1 from hBMSCs, hUVECs, and hUASMCs in different systems. **c** Expression of TβRII in hUVECs and hUASMCs induced by TGFβ3 assessed by western blot analysis. **d** Expression of p-Smad3 and Smad3 in hUVECs and hUASMCs induced by TGFβ3 assessed by western blot analysis. **P < 0.01, ***P < 0.005, ****P < 0.001. hUASMC human umbilical artery smooth muscle cell, hUVEC human umbilical vein endothelial cell, MSC mesenchymal stem cell, TGFβ3 transforming growth factor beta-3

The article "TGFβ3 recruits endogenous mesenchymal stem cells to initiate bone regeneration" was retracted in 2022. Reasons: duplicated images; original data or images not available; unreliable results or conclusions.

### Vascular cells secreted MCP1 accompanied by the activity of TβRII/Smad3 signaling

TGFβ1 has been reported to induce MCP1 expression in A375 human melanoma cells and vascular smooth muscle cells by Smad3, whereas TGFβ1 downregulates MCP1 expression in macrophages via inhibition of Smad3 [32–34]. These studies suggest that Smad3 is the essential effector for MCP1 expression remediated by TGFβ1. To date, TGFβ3 has rarely been reported to promote MCP1 in hUASMCs or hUVECs. According to the aforementioned studies, the mechanism of TGFβ3-induced MCP1 in vascular cells should focus on the Smad3 signaling pathway. TGFβ3 stimulation could enhance the expression of TβRII and p-Smad3 in hUASMCs and hUVECs, but not Smad3 (Fig. 3c, d). The expression of TβRII in hUASMCs and hUVECs increased 112.0 ± 10.5% and 132.9 ± 9.3% against the nonstimulation, respectively (*P* < 0.001 for hUVECs, *P* < 0.005 for hUASMCs; Fig. 3c). Accordingly, the expression of p-Smad3 in hUASMCs and hUVECs increased 46.0 ± 6.7% and 129.1 ± 9.5% relative to the nonstimulation, respectively (*P* < 0.001; Fig. 3d).

### Knockdown of Smad3 in vascular cells inhibited TGFβ3-induced hBMSC migration

Smad3 phosphorylation played an important role in TGFβ1-induced MCP1 secretion [33]. To determine whether knockdown of Smad3 in vascular cells affects TGFβ3-induced hBMSC migration in the coculture system, Smad3 siRNA was transfected to vascular cells, and the expressions of Smad3 decreased 70.8 ± 1.4% and 80.8 ± 2.2% in hUASMCs and hUVECs compared to scrambled ones, respectively (*P* < 0.001; Fig. 4a, b). Knockdown of Smad3 also decreased MCP1 secretion by 57.2 ± 3.6% and 56.7 ± 3.7% in hUASMCs and hUVECs, respectively (*P* < 0.001; Fig. 4c). In the coculture system, vascular cells with knockdown of Smad3 decreased the number of migrated hBMSCs (Fig. 4d). The number of migrated hBMSCs in the Smad3 siRNA hUASMC and Smad3 siRNA hUVEC groups decreased 52.5 ± 4.0% and 56.7 ± 3.8% compared to the scrambled hUASMC and scrambled hUVEC groups (*P* < 0.001; Fig. 4d).

**Fig. 4:** Knockdown of Smad3 in vascular cells inhibited TGFβ3-induced hBMSC migration. **a** Expression of Smad3 in hUVECs and hUASMCs were transfected with *siRNA Smad3* as assessed by western blot analysis. **b** Relative density of Smad3 for (**a**). **c** Secretion of MCP1 in different cells. **d** Transwell assay for hBMSC migration in the coculture system of hBMSC and vascular cells with or without knockdown of Smad3. Migrated cells were stained purple with crystal violet. Scale bar: 100 μm. **P < 0.01, ****P < 0.001. hUASMC human umbilical artery smooth muscle cell, hUVEC human umbilical vein endothelial cell, MSC mesenchymal stem cell, siRNA small interfering RNA, TGFβ3 transforming growth factor beta-3

The article "TGFβ3 recruits endogenous mesenchymal stem cells to initiate bone regeneration" was retracted in 2022. Reasons: duplicated images; original data or images not available; unreliable results or conclusions.

### TGFβ3 recruited endogenous MSCs to initiate bone formation

To assess whether TGFβ3 could promote the recruitment of host MSCs, the scaffolds loading 1 μg TGFβ3 were prepared with absorbable gelatin sponges by physical adsorption. At 3 days post implantation, TGFβ3 delivery induced an increase in MCP-1 level by 7.9 ± 1.1-fold compared with the TGFβ3-free cells (*P* < 0.001 for TGFβ3 group vs vehicle group; Fig. 5a). Based the result of Fig. 3b showing that MCP1 was mainly secreted from vascular cells, upregulation of the MCP1 level in vivo might maintain a close relationship with an increase in the number of vascular cells recruited by TGFβ3 (*P* < 0.01; Fig. 5b, c). Sections of the TGFβ3 group showed darker positive staining of CD31 than the TGFβ3-free group and the CD31^+^ vascular cells in the TGFβ3 group formed into a circle of vascular lumen, but not those in the TGFβ3-free group (Fig. 5b). Furthermore, TGFβ3 delivery also recruited 201.5 ± 9.6% CD31^+^ vascular cells relative to the TGFβ3-free group at 7 days post implantation (*P* < 0.01; Fig. 5b, c).

**Fig. 5:** TGFβ3 recruited endogenous MSCs to initiate bone formation. **a** Expression of MCP1 in regenerated tissue in the TGFβ3 and vehicle groups at 3 days post implantation. **b** Immunohistochemical analysis for CD31^+^. Scale bar: 100 μm. **c** Number of CD31^+^ cells. **d** Immunofluorescent images of Sca-1 and PDGFR-α in scaffolds; green, Sca-1; red, PDGFR-α; blue, DAPI. Scale bar: 20,000 nm. White arrows, Sca-1^+^ PDGFR-α^+^ MSCs. **e** Recruited MSC%. **f** 3D and 2D center-sagittal view images of regenerated bone mass in the TGFβ3 and vehicle groups at 8 weeks post implantation. Scale bar: 10 mm. **g** BV/TV and BMD of the regenerated bone in (**f**). *P < 0.05, **P < 0.01, ****P < 0.001. BMD bone mineral density, BV/TV bone volume fraction, MCP1 monocyte chemotactic protein 1, MSC mesenchymal stem cell, TGFβ3 transforming growth factor beta-3

More vascular cells and a higher level of MCP1 resulted in much more MSCs. Colonization by host cells was evident in the TGFβ3 group and to a lower extent in the vehicle group (blue DAPI staining) at 7 days post implantation. The amount of homing MSCs, colabeled with green Sca-1 staining and red PDGFR-α staining, in TGFβ3 constructs were more than that of vehicle constructs at 7 days post implantation (Fig. 5d). TGFβ3 delivery recruited approximately 191.4 ± 7.4% MSCs relative to spontaneous MSC migration without TGFβ3 (*P* < 0.01; Fig. 5e). Furthermore, TGFβ3-induced homing of MSCs to the defect site remarkably achieved a great amount of new bone tissue, in strong contrast to the vehicle administration did, which was shown by the segmentation of micro-computerized tomography images (Fig. 5f). Last, the amount of mineralized tissue from micro-CT results was quantified. TGFβ3 delivery achieved 259.1 ± 17.0% BV/TV and 190.0 ± 12.5% BMD compared with those of the vehicle group at 8 weeks post implantation (Fig. 5g).

The article "TGFβ3 recruits endogenous mesenchymal stem cells to initiate bone regeneration" was retracted in 2022. Reasons: duplicated images; original data or images not available; unreliable results or conclusions.

## Discussion

MSC recruitment underlies the regeneration of bone tissue in vivo [1]. The mode of recruitment used in tissue regeneration is directional migration in response to chemokines [5]. TGFβs include three different isoforms (TGF-β1, TGF-β2, and TGF-β3), and TGFβ1 has been considered a major factor that regulates osteoblasts and osteoclasts in bone homeostasis [30, 35]. TGFβ2 and TGFβ3 levels increased in the chondrogenesis occurring during fracture healing [36]. Thus, most studies focus on the effect of TGFβ1 on MSC recruitment for bone regeneration, while TGFβ3 is examined for its potential role in cartilage regeneration. The present study reports that TGFβ3 could recruit MSCs to initiate bone regeneration (Fig. 5). We demonstrated that TGFβ3 could directly increase the migrated hBMSC by 39%, which is rarely reported (Fig. 1). Zhang et al.’s [33] studies showed that TGFβ1 had no direct effect on BMSC migration. The data showed that TGFβ3 has superior promigratory properties on BMSCs to TGFβ1. MSCs are recruited to locations by homing through the vascular network [9, 14]. In the present study, hUASMCs or hUVECs could alone improve hBMSC migration, in which hUVECs enhanced approximately 1.4-fold the number of migrated cells relative to hUASMCs (Fig. 2). Furthermore, in the coculture system of hBMSCs and hUVECs, the low concentration of TGFβ3 administration enhanced cell mobilization by approximately 52% (Fig. 2). Our data followed a similar trend to the findings of Zhang et al. [33], in which their studies showed that TGFβ1 promotes MSC migration by rat vascular smooth muscle cells. These results showed that TGFβ3 promoted migration of hBMSCs in direct and indirect manners and indirect manner caused the greater amount of migrated MSCs. Finally, in-vivo immunofluorescent images of endogenous MSC homing verified that the chemotaxis of MSCs can be enhanced by TGFβ3 (Fig. 5b).

A few studies have shown increasing evidence for a link between bone metabolism and the vasculature; that is, the so-called “bone-vascular axis” [31, 37, 38]. In the present study, TGFβ3 not only recruited MSCs, but also recruited vascular cells. TGFβ3 delivery can induced 200% CD31^+^ vascular cell homing, accompanied with a striking 7.9-fold increase of MCP1 in contrast to the TGFβ3-free group, which has been reported to be involved in the recruitment of stem/progenitor cells to the vasculature (Fig. 5a) [11]. According to the result that MCP1 was secreted from vascular cells, not from hBMSCs in vitro, we can infer that TGFβ3-recruited vascular cells improved endogenous MSC homing by MCP1 secreted by vascular cells (Fig. 3). These results explain why endogenous MSCs might move to the vasculature during injury. Furthermore, TGFβ3 recruited a greater amount of MSCs, and achieved the better bony bridging of the defects than TGFβ3-free did (Fig. 5).

The article "TGFβ3 recruits endogenous mesenchymal stem cells to initiate bone regeneration" was retracted in 2022. Reasons: duplicated images; original data or images not available; unreliable results or conclusions.

The specific receptors of the isoform TGFβ3 are TβRII/I, as the specific receptors of the TGFβ superfamily, which have been demonstrated to be expressed in many types of cells, including MSCs and vascular cells ([15, 39, 40]). In the present study, TGFβ3 directly enhanced hBMSC migration by 39% via upregulation of the expression of TβRII, while blocking the TGFβ signaling pathway resulted in ineffectiveness of TGFβ3 stimulation (Fig. 1). In the coculture system of hBMSCs and vascular cells, the almost 60% MCP1 level and MSC migration can be inhibited via knocking down Smad3 to block the TGFβ signaling pathway in vascular cells (Fig. 4). In vivo, upregulating MCP1 to increase MSC homing, as well as to enhance bone formation, verified that the TGFβ3 signaling pathway played an important role in recruiting MSC to initiate bone regeneration (Fig. 6).

**Fig. 6:** Schematic representation of the direct and indirect mechanism of TGFβ3-induced MSC migration based on this study. Black arrow, direct mechanism; red arrow, indirect mechanism. MCP1 monocyte chemotactic protein 1, MSC mesenchymal stem cell, Tgfbr1 TGFβ type I, Tgfbr2 TGFβ type II, TGFβ3tTransforming growth factor beta-3

## Conclusions

We demonstrated that TGFβ3 could not only directly improve the migration of hBMSCs through the TGFβ signaling pathway but could also upregulate the secretion of MCP1 from vascular cells in a Smad3-dependent manner, which heavily amplified the promigratory capacity of TGFβ3 on hBMSCs. Moreover, TGFβ3 delivery recruited many more Sca-1^+^PDGFR-α^+^ MSCs via increasing MCP1 secretion to initiate bone regeneration. Previous studies have typically focused on the role and mechanism of TGFβ3 in cartilage regeneration, while from a novel perspective the present study demonstrated that TGFβ3 recruited and instructed endogenous MSCs toward bone formation mediated by vascular cells. This may shed light on the improvement of MSC homing in bone regeneration.

The article "TGFβ3 recruits endogenous mesenchymal stem cells to initiate bone regeneration" was retracted in 2022. Reasons: duplicated images; original data or images not available; unreliable results or conclusions.

## Abbreviations

hBMSC: Human bone marrow MSC
hUASMC: Human umbilical artery smooth muscle cell
hUVEC: Human umbilical vein endothelial cell
MCP1: Monocyte chemotactic protein 1
MSC: Mesenchymal stem cell
siRNA: Small interfering RNA
TβRI: TGFβ type I receptor
TβRII: TGFβ type II receptor
TGFβ3: Transforming growth factor beta-3
